# NUT Midline Carcinoma: A Rare Solid Tumour Characterized by Chromosome Rearrangement

**DOI:** 10.1155/2022/3369895

**Published:** 2022-07-04

**Authors:** Huan Zhang, Weili Kong, Wei Liang

**Affiliations:** ^1^Department of Oncology, The Third Affiliated Hospital of Chongqing Medical University, Chongqing 401120, China; ^2^Department of Otorhinolaryngology Head and Neck Surgery, West China Hospital, Sichuan University, Chengdu 610041, Sichuan, China

## Abstract

**Objective:**

Rare and poorly differentiated NUT midline carcinoma (NMC) is a highly malignant tumour. However, due to the rarity of NMC, reports on its clinical, imaging, and pathologic features are still scarce.

**Methods:**

In this study, three patients diagnosed with NMC located in the parotid gland, lung, and trachea were used as examples to summarize the clinicopathological features of NMC. All the cases were diagnosed by measuring positive nuclear reactivity to NUT antibody after dual-colour FISH tests were conducted, and all of the results were positive, indicating chromosomal rearrangements on 15q14 of the NUT gene.

**Results:**

These three patients were treated with conventional treatments, including surgical therapy and chemoradiotherapy. Given the poor efficacy of intensive conventional treatment, two novel therapies, histone deacetylase inhibitors (HDACi) and bromodomain inhibitors (BETi) are recommended, as both can arrest the growth of tumour cells, and these targeted therapies may extend patient survival time in the future.

**Conclusions:**

NMC is an easily misdiagnosed cancer with a poor prognosis; therefore, improving the awareness of clinicians is critical for increasing the diagnostic accuracy, and selecting effective treatment is the main method to improve prognosis.

## 1. Introduction

Nuclear protein in testis (NUT) midline carcinoma represents a rare, poorly differentiated, and highly malignant solid tumour characterized by translocations involving the NUT gene which can be detected by FISH and PCR on chromosome 15q14 [1]. It is commonly reported that the NUT fusion genes in NMC include BRD4-NUT fusion gene caused by translocation t(15;19)(q14;p13.1), BRD3-NUT fusion gene caused by translocation t(9;15)(q34.2;q14), NSD3-NUT fusion gene caused by translocation t(8;15)(p11.23;q14) [2,3]. Uncommonly, a unique cytogenetic abnormality of three-way translocations has been reported in NMC, including t(4;15;19) [4], t(9;15;19) [5], t(11;15;19) [6], and t(2;9;15) [2].

Most squamous cell carcinomas are the result of complex and multiple genetic abnormalities, and very few are caused by chromosome rearrangement. The mechanism of the BRD4-NUT fusion oncogene was first identified in an epithelial tumour in 2003 [7]. So far, at least 63 cases diagnosed as NMC have been reported [8]. The name NUT midline carcinoma is designated for this malignancy because the primary tumour in most cases arises from midline anatomic structures in the head and neck, chest (including the nasal cavity, sinus, nasopharynx, epiglottis, larynx, mediastinum, and lung) [9,10]. In addition, other tumour locations, including the kidney, bladder, and iliac bone, have been reported [11,12]. The previously reported literature has shown that NMC can equally affect individuals at any age (0-78 years, median 16) and both sexes with a slight female predominance in the incidence with a ratio of 1.5 : 1 [13].

The BRD4-NUT fusion oncogene blocks squamous cell differentiation and promotes NMC cell growth, while most NMC pathology specimens exhibit abrupt focal squamous differentiation [12]. Some researchers hold the viewpoint that NMC is a subtype of squamous cell carcinoma because of the morphological characteristics of undifferentiated or poorly differentiated carcinoma with focal squamous differentiation. Apart from specialized genetic testing, immunohistochemical staining of NUT-1, a monoclonal antibody, has been considered as the diagnostic criterion with 100% specificity and 87% sensitivity [14].

So far, there is no specific treatment for NMC. Despite conventional therapies such as surgery and chemoradiotherapy, whether in young patients or elderly patients, the prognosis of NMC is extremely poor, with a median overall survival of 6.7 months [15]. Therefore, it is vital to develop targeted therapeutics. There are two kinds of novel agents, histone deacetylase inhibitors (HDACi) and BET inhibitors, currently in clinical trials [8].

Although there have been three cases of NMC with different primary sites identified in this institute, a larger series describing NMC is essential. Due to the rarity and poor prognosis of NMC, it is essential to know more about it. The purpose of this article is mainly to provide the clinicopathological features of NUT midline carcinoma so that a high level of suspicion for NMC is expected to be maintained by clinicians when these features are present.

## 2. Materials and Methods

### 2.1. Case Series

This study was approved by the Research Ethics Board of West China Hospital (WCH), and pathology records were collected. A total of 3 cases were identified under the testing results “immunohistochemical stain positive for NUT” associated with a biopsy or operation specimen procured from any site (including head and neck, chest, abdomen, and bone tissues). Pathology slides of all cases were reviewed in WCH archives, patient information, treatment process, and examination results were derived from the electronic medical records.

### 2.2. Laboratory Tests

Laboratory tests, including blood routine, stool routine, urine routine, liver and kidney function, and electrocardiogram, were performed for the three patients mentioned above.

### 2.3. Radiology Tests

All patients underwent chest computed tomography (CT) scans, head and neck magnetic resonance imaging (MRI), abdominal CT, and bone scintigraphy. All imaging findings were reviewed to identify the primary and metastatic sites.

### 2.4. Immunohistochemistry

IHC was performed as described previously [9]. anti-NUT (C52B1) rabbit mAb (1 : 200, CST, Inc.). IHC staining for NUT was interpreted by experienced pathologists. Tumour specimens in the three cases were stained for P63, CK5/6, P40, TTF-1, NapsinA, PCK, Syn, CgA, Ki-67, ROS-1, ALK-V, and PDL1.

### 2.5. Fluorescence in Situ Hybridization

As previously described, chromosomal translocation of the NUT gene locus was performed by FISH in NUT-IHC-positive cases [9]. The SPEC NUTM1 Dual Colour Break Apart Probe, a mixture of two direct-labelled probes hybridizing to the 15q14 band, was used to detect translocations involving the chromosomal region 15q14 harbouring the NUTM1 gene. The green fluorochrome direct-labelled probe hybridizes proximal to and the orange fluorochrome direct-labelled probe hybridizes distal to the NUTM1 gene. With the use of appropriate filter sets, green and orange hybridization signals appeared in the labelled chromosomal region 15q14. In interphases of normal cells or cells without a translocation involving the 15q14 band, two green/orange fusion signals are detected. One 15q14 locus affected by a translocation is indicated by one separate green signal and one separate orange signal.

## 3. Results

The information of three patients diagnosed with NMC are listed in Tables 1–3.

### 3.1. Clinical Findings

According to the clinical history in Table 1, the mean age of the patients at the time of diagnosis was 32 years old (ranging from 21 to 41). They had no history of smoking, drinking, drug abuse, or radiation exposure, and no significant past medical history. In addition, all these patients were men, and their parents and siblings were healthy without any known family history of malignancy. The primary sites of these three cases were the parotid gland, right lung middle lobe, and lower trachea.

The first patient presented a history of a painful lump below the left ear, which was the parotid gland. The second patient complained of back pain caused by tumour invasion. The third patient complained of cough and haemoptysis, which are commonly seen in lung cancer. The results of the routine blood counts and liver, kidney, and coagulation functions were normal in all patients. Thus, all clinical symptoms were caused by tumour cell infiltration, transfer, diffusion, and oppression.

### 3.2. Imaging Findings

Imaging data were available for review in electronic documents from the Imaging Department (Table 2). In Case 1, the primary mass was in the parotid gland. A CT scan of the parotid gland revealed an enlarged, substantially inhomogeneous mass with an unclear border in the left parotid gland (Figure 1(a)), consistent with the radiological features of parotid gland malignant tumours. Two months after the first stage of therapy, the patient presented to the institute with a progressive headache, ptosis of the left eye, eye movement disorder, and visual impairment. Enhanced MRI of the sella turcica region revealed a soft tissue mass involving the nasopharynx, pituitary, left cavernous sinus, and meninges, which explained the symptoms caused by tumour invasion, causing optic nerve damage and skull base destruction.

In case 2, the patient presented to the outpatient department with a 2-month history of back pain accompanied by lower limb weakness and difficulty relieving the bowels. A chest CT scan revealed a lobulated soft mass with a vague margin of approximately 4.3 × 3.5 cm located in the right middle lobe lung accompanied by stenosis in the local lumen, leading to atelectasis of the right middle lobe, enlarged hilar lymph nodes, enlarged mediastinal lymph nodes, and diffusing nodules in the bilateral pulmonary region, all of which were considered metastatic lesions (Figure 1(b)). Enhanced magnetic resonance imaging (MRI) of the thoracic vertebra showed multiple vertebral bone destruction. The imaging features of the lung NUT midline carcinoma were extraordinarily similar to those of lung cancer.

In case 3, a chest CT scan showed a mass with an irregular shape located in the bifurcation of the trachea (Figure 1(c)), which explained the chief complaint of haemoptysis. From the information above, it can be concluded that there are no special characteristic imaging features of NUT midline carcinoma.

### 3.3. Pathologic Findings

The pathologic features are recorded in Table 3. The three patients were admitted with different presumptive diagnoses, including poorly differentiated squamous cell carcinoma and central lung cancer. The pathology reports of the three cases all described a neoplasm formed by nests of poorly differentiated cells with abrupt areas of squamous differentiation (Figure 2). The poorly differentiated tumour cells showed positive immunoreaction to NUT antibody and P63, CK, and P40 (Figure 3). All tumours showed positive expression of squamous cell carcinoma markers, such as positive P63, and negative expression of adenocarcinoma markers, such as TTF1.

Immunohistochemical analysis for NUT was performed with anti-NUT (C52B1) rabbit mAb, IHC staining for NUT proved to be positive when there is a strong, speckled nuclear staining in greater than 50% of nuclei (Figure 4). In addition, FISH testing was performed on all cases to determine the chromosome translocation, and the NUT fusion oncogene was found in all cases (Figure 5). These results showed that NMC had similar characteristics to poorly differentiated squamous carcinoma. By NUT mAb testing or FISH testing, the diagnosis of NMC was confirmed.

### 3.4. Treatment and Outcomes

In Case 1, considering that the lump might be a tumour, the patient received total parotidectomy and 2 cycles of chemotherapy (chemotherapy regimen included paclitaxel and cisplatin) followed by radiotherapy, as the tumour was confirmed to be malignant by postoperative pathology.

Two months after the first stage of treatment, the patient presented to the institute with progressive headache, ptosis of the left eye, eye movement disorder, and visual impairment. Skull base and nasopharyngeal region metastasis of the tumour was confirmed by enhanced MRI of the head and nasopharyngeal laryngoscope. The immunohistochemical staining of the nasopharyngeal mucosa revealed the positivity of NUT, proving it to be a NUT carcinoma.

Therefore, the patient received 1 cycle of chemotherapy followed by intensity-modulated radiotherapy while the chemotherapy regimen included gemcitabine and cisplatin. At the 4-month follow-up, no recurrence or metastasis was detected.

In case 2, the patient was diagnosed with distant metastasis on the initial visit. The primary site was in the right lung middle lobe, and imaging examination confirmed metastatic lesions in the bilateral pulmonary, hilar lymph nodes, mediastinal lymph nodes, and multiple thoracic vertebrae. The immunohistochemical staining of the right lung mass revealed positivity for NUT, confirming the diagnosis of NUT midline carcinoma.

The patient received radiotherapy to the thoracic vertebra to relieve pain before leaving the hospital without any further treatment because of financial difficulties. The patient died within 1 month after being discharged.

In case 3, the patient received resection of the tracheal tumour after the CT scan of the chest, demonstrated a mass in the lower trachea. However, a recurrence occurred within one month. From these three cases, NMC was found to be a highly aggressive carcinoma with a high incidence of recurrence and metastasis.

## 4. Discussion

In this study, complete clinical, radiographic, and pathologic details for the three patients diagnosed with NMC are provided. Combined with the previously reported literature, no specific risk factors for NMC were found. All the patients complained about local symptoms caused by tumour oppression and diffusion. In addition, there were no special characteristic imaging features, and NMC could be misdiagnosed as a poorly differentiated squamous cell carcinoma due to the difficulty of distinguishing it morphologically from non-NMC poorly differentiated squamous cell carcinoma.

As described above, the patients were initially misdiagnosed as poorly differentiated squamous cell carcinoma based on pathological biopsy, after which the diagnosis was revised to NMC based on IHC staining for NUT as well as FISH. Previously, the diagnostic criteria of NMC is karyotype analysis demonstrating the chromosomes rearrangement result in t(15;19) (q14,p13.1) [16]. The invention of the BRD4-NUT fusion oncogene by FISH has made the detection of NMCs quickly and accurately, and all NMCs can be detected, including all NUT variants. Recently, the IHC test for NUT with high sensitivity and specificity has simplified the diagnosis greatly. The only other tumours that could display nuclear NUT reactivity are germ cell tumours with a focal (<5%), faint, and lack of speckled pattern staining [17]. Therefore, FISH, RT-PCR, or karyotype analysis is no longer required for diagnosis since the specificity of the NUT antibody is 100% with a sensitivity of 87% [17]. Although these conventional diagnostic methods are not necessarily required for the diagnosis, determination of the specific fusion is recommended because this may influence treatment decisions.

It is extremely difficult for pathologists to diagnose NMC based on morphology, and the greatest challenge is the uncertainty of when to test for it. There are some features that may help in the recognition of this tumour and guide further diagnostic examinations. One unique feature is that the cells vary from small to medium in size with a conspicuously monotonous appearance, but there are often areas of focal “abrupt” squamous differentiation while the rest of the tumour appears to be mostly poorly differentiated [17]. In these cases, pathologists should have a high suspicion of NMC and perform further examinations, such as immunohistochemical tests for NUT, FISH, RT–PCR, or karyotype analysis.

In this study, the patients were treated with conventional treatments, including surgical therapy and chemoradiotherapy. In Case 1, the patient who received surgical therapy and chemoradiotherapy achieved an overall survival of 14 months (Table 1), a better treatment effect than the other two patients. By reviewing previous literature, different chemotherapy regimens were found to have been used to treat patients with NMC, and these chemotherapy regimens included platinum, taxanes, anthracyclines, and nonplatinum alkylating agents [5,8,15]. However, no chemotherapeutic regimen exists for NUT carcinoma. In a retrospective study of 54 patients diagnosed at NMCs with different primary sites, multivariate analysis suggested that the extent of surgical resection and initial radiotherapy were independent predictors of PFS and OS, and the median overall survival was 6.7 months [15]. In another retrospective study of 48 patients whose diagnoses were head and neck NMCs, aggressive initial surgical resection with or without postoperative chemoradiation or radiation was proven to be associated with significantly enhanced survival, and the median overall survival was 9.7 months [8]. In a recent retrospective study of 8 primary pulmonary NMCs, despite chemotherapy or chemoradiotherapy, the median overall survival was 2.2 months [9]. Therefore, it can be inferred that the primary sites may be independent prognostic factors, and thoracic involvement and metastatic spread may be associated with shorter overall survival.

A combination of surgical resection and chemoradiotherapy can be considered the main regimen in the treatment of NMC. However, most patients are not able to achieve long-term survival, and the situation may be worse when they are diagnosed with distant metastasis. Therefore, it is essential to find a more effective and safer treatment protocol. A novel therapy is under investigation, where two molecular-targeted drugs aimed at the underlying pathogenic mechanism have emerged. They are bromodomain inhibitors (BETi) and histone deacetylase inhibitors (HDACi), both of which can induce differentiation and arrest the growth of NMC cells.

As described above, the mechanism of NMC is the function of the BRD4-NUT protein, which causes tumour cell proliferation and prevents cellular differentiation. Silencing RNA (siRNA) has been used to demonstrate that knockdown of BRD4-NUT in NMC cells results in growth arrest and prompt terminal squamous differentiation [18]. As such, BETis could inhibit the function of the BRD4-NUT protein, allowing cellular differentiation to proceed. As indicated in one study, after taking a novel oral BET inhibitor named OTX015/MK-8628, which is able to target BRD2/3/4/T with impressive preclinical and rapid antitumour activity against NMC, two patients achieved notably longer overall survival (19 and 18 months, respectively) than the median survival of 6.7 months reported in the largest retrospective series of patients with NMC [18].

The BRD4-NUT oncoprotein can bind and activate histone acetyltransferase, which leads to the acetylation of chromatin and creates a feed-forward mechanism leading to neoplasia. Histone deacetylase inhibitors (HDACis) artificially increase acetylation, leading to BRD4-NUT function reversal and thus a return to regular cellular progression [19].

Dual PI3K and HDAC inhibition by CUDC-907 shows remarkable single-agent activity and a strong synergistic effect with PARP inhibitor olaparib in SCLC [20]. According to the International NMC Registry (https://www.nmcregistry.org), a clinical trial investigated the use of a recommended phase 2 dose of CUDC-907, a dual PI3 kinase/HDAC inhibitor drug, which was proven to have potent activity against NMC cells. Clinical trials used to evaluate the efficacy of either HDACi or BETi may eventually confirm the effect in treating NMC.

To date, no effective treatment exists for NMC, and surgical resection and radiochemotherapy are obviously not enough to achieve good survival. Two promising therapies, HDACi and BETi, are currently under study, and perhaps they will improve the outcome of these patients in the future.

## Figures and Tables

**Figure 1:** Parotid gland CT scan revealed an enlarged, substantially inhomogeneous left parotid gland with an unclear border mass (a). Chest CT scan revealed a lobulated soft mass with a vague margin located in the right lung middle lobe accompanied by stenosis of the local lumen leading to atelectasis of the right middle lobe (b). Chest CT scan also showed an irregularly shaped mass located in the bifurcation of the trachea (c).

**Figure 2:** Histomorphology of NUT midline carcinoma (case 3): poorly differentiated tumour cells and focal keratinization (H&E stain, ×40) (a). Higher magnification shows that most of the cells were incohesive, monotonous, atypical, and scanty-cytoplasm tumour cells with irregular ovoid hyperchromatic nuclei (H&E stain, ×400) (b).

**Figure 3:** Immunohistochemical staining for P63 (a) and CK (b) in case 3: positive reactivity in the tumour cells.

**Figure 4:** Immunohistochemical staining for NUT (case 3): strong and diffuse nuclear reactivity of NUT in the tumour cells (200×).

**Figure 5:** Fluorescence in situ hybridization testing: two orange/green fusion signals represents two normal (nonrearranged) 15q14 loci. A signal pattern consisting of one orange/green fusion signal, one orange signal, and a separate green signal indicates one normal 15q14 locus and one 15q14 locus affected by a translocation. An NMC tissue section with a translocation of the NUTM1 gene is identified by one nonrearranged orange/green fusion signal, one orange and one separate green signal, which indicates the translocation ((a) case 1, (b) case 2, (c) case 3).

**Table 1:** Clinical features of patients diagnosed with NUT midline carcinoma.

Case	Age	Sex	Tabacco history	Presenting symptoms	Primary site	Metastasis sites	Treatment	Survival time
1	21	M	Never	Painful lump below the left ear ×3 months	Parotid gland	Nasopharynx cavernous sinus skull base meningeal	Surgical treatment chemotherapy radiotherapy	Longer than 14 months

2	41	M	Never	Back pain ×2 months	Right lung middle lobe	Hilar lymph nodes mediastinal lymph nodes bilateral pulmonary multiple thoracic vertebra	Radiotherapy for thoracic vertebra	1 Month

3	34	M	Never	Productive cough, haemoptysis ×3 weeks	Lower trachea	No metastasis was found at first diagnosis	Surgical treatment	3 Months

**Table 2:** Radiographic features of NUT midline carcinoma.

Case	Primary sites	Size (imageology)	Features	Metastasis sites	Lymphadenopathy	Size (surgical specimen)
1	Parotid gland	Approximately 3 × 2.1 cm	Substantially inhomogeneous Unclear border	Nasopharynx Cavernous sinus Skull base Meningea	Enlarged cervical lymph node	4 × 3 × 3 cm

2	Right lung middle lobe	Approximately 4.3 × 3.5 cm	Lobulated Unclear border	Bilateral pulmonary	Enlarged hilar lymph nodes Enlarged mediastinal lymph nodes	No surgical specimens

3	Lower trachea	Approximately 3.9 × 3.5 cm	Substantially inhomogeneous Unclear border	No metastasis was found at first diagnosis	No enlarged lymph nodes	4 × 3 × 3 cm

**Table 3:** Pathologic features of NUT midline carcinoma.

Case	Biopsy sites	Under naked eye	Presumptive diagnosis	Squamous cell carcinoma expression	Adenocarcinoma maker expression	Neuroendocrine marker expression	Target detection	NUT IHC result	Fish result
1	Nasopharyngeal region	Hard	Poorly differentiated squamous cell carcinoma	P63(+)CK5/6(+) P40(partially+)	TTF-1(-)	Not detected	Not detected	Positive	NUT fusion oncogene
2	Lung tumour	No vision of surgical field	Central lung cancer	P63(+) P40(+)	TTF-1(-)	Syn(-) CgA(-) Ki-67 (60%)	ROS-1(-) ALK-V(-) PDL1(+,100%)	Positive	NUT fusion oncogene
3	Tracheal tumour	Hard Unclear border fish flesh appearance	Poorly differentiated squamous cell carcinoma	P63(+) P40(+)	TTF-1(-) NapsinA(-)	Not detected	ROS-1(-) ALK-V(-) PDL1(-)	Positive	NUT fusion oncogene

## Data Availability

The data that support the findings of this study are available on request from the corresponding author.
